The article "Intelligent Internet of Things Medical Technology in Implantable Intravenous Infusion Port in Children with Malignant Tumors" was retracted in 2023. Reasons: signs of a paper mill; suspected computer-generated content; unreliable results or conclusions; lack of ethics approval or compliance.

# Intelligent Internet of Things Medical Technology in Implantable Intravenous Infusion Port in Children with Malignant Tumors

**DOI:** 10.1155/2021/8936820

**Published:** 2021-11-28

**Authors:** Shaohong Liu, Luxing Jiang, Xin Wang

**Affiliations:** Department of Pediatric Surgery, Hunan Children's Hospital, Changsha 410007, China

## Abstract

Due to the recent technological revolution that is centered around information technology, the Internet of Medical Things (IoMT) has become an important research domain. IoMT is a combination of Internet of Things (IoT), big data, cloud computing, ubiquitous network, and three-dimensional holographic technology, which is used to build a smart medical diagnosis and treatment system. Additionally, this system should automate various activities, such as the patient's health record and health monitoring, which is an important issue in the development of modern and smart healthcare system. In this paper, we have thoroughly examined the role of a smart healthcare system architecture and other key supporting technologies in improving the health status of both indoor and outdoor patients. The proposed system has the capacity to investigate and predict (if feasible) the clinical application and nursing effects of totally implantable intravenous port (TIVAP) in pediatric hematological tumors. For this purpose, seventy children with hematologic tumors were treated with TIVAP, and IoMT-enabled care was provided to them, where the occurrence of adverse events, specifically after the treatment, was observed. The experimental results collected after the 70 children were treated and cared for by TIVAP show that there were five cases of adverse events, whereas the incidence rate of the adverse events was 7.14%. Moreover, TIVAP has significant efficacy in the treatment of hematologic tumors in children, and it equally reduces the vascular injury caused by chemotherapy in younger patients. Likewise, targeted care reduces the incidence of adverse events in children with expected ratio.

## 1. Introduction

A serious and challenging issue to the health of individuals is generated because of the current industrialization, urbanization, population aging, changing disease spectrum, and ecological changes. Additionally, a smart healthcare system has various problems such as rapid cost growth, poor accessibility, uneven resource allocation, inefficient services, and uneven service quality. To cope with these problems, an intelligent medical or Internet of Medical Things (IoMT) network was introduced in the literature [1, 2]. With the development and implementation of the internet and “Belt and Road” formation strategy, new technologies, such as the Internet of Things (IoT), big data, cloud computing, ubiquitous networks, and three-dimensional holographic technology, were introduced. They have a significant impact on the concept, model, technology, and methods of medical services or activities. Today, with the increasing concentration of data, medical boilers are increasingly relying on the internet or business networks to extend their services to the streets, communities, enterprises, and families [3, 4].

In foreign countries, the smart healthcare domain is assumed to be a mature research field and is efficiently utilized in the smart healthcare system to automate various activities that are tightly coupled with patients and doctors. The Institute of Medicine of the United States (IOMI991) has developed a prototype of intelligent medical care. It has the capacity to automate various activities with available resources in the hospitals, such as the electronic medical records that exist in a special system. It provides support to its users to obtain complete and accurate information. Also, it provides alerts to the medical personnel and various medical decision support systems. In 2004, Japan's Ministry of Internal Affairs and Communications (MC) held a policy forum on the realization of a ubiquitous network society and proposed the “u-Japan strategy.” In 20l1, Japan's strategic headquarters and the Ministry of Internal Affairs and Communications (MC) proposed the concept of “My Hospital Everywhere,” [5, 6] where the individuals are able to not only obtain medical and health information from the medical institutions but also maintain and manage information through smart terminals, such as computers. For the convenience of patients, Japan plans to implement a seamless community cooperative medical service that provides access to medical and nursing services from different medical institutions, regions, and specialties.

Intelligent medical care is still in the preliminary stage, particularly in China, and it is moving from clinical automation to regional automation. The Health and Welfare Commission has formulated corresponding policy plans after the pilot work of regional healthcare repository in Shanghai and Guangdong [7–9]. We should vigorously support the construction of information technology and resource integration in medical treatment, health care, medicine, medical insurance, financial supervision, and so on. The standardization of medical information and the construction of public service information platforms have laid the foundation for the realization of a unified, efficient, and interconnected smart medical platform. Beijing, Shanghai, Wuhan, and other cities have recently initiated a construction plan and the concept of smart medical healthcare system, which are expected to benefit the people in the future [10].

The implacable intravenous port, which is medically known as a port, is shown in Figure 1. It is a novel infusion method to facilitate long-term infusion. It is more common in western developed countries and is now becoming popular in most parts of China. It mainly consists of an injection seat, a catheter, and a butterfly needle. After the subcutaneous implantation of the injection seat, the catheter inserted into the central vein is connected to establish long-term vascular access, which can play a role similar to that of a port, and hence, the name infusion port. It is suitable for long-term or repeated drug administration, infusion of highly concentrated chemotherapy drugs, parenteral nutrition solution, blood transfusion, blood sample collection, etc. [11]

The advantages of an implacable IV port are as follows: (i) it is implanted once, (ii) it reduces the pain and difficulty of repeated punctures, and (iii) the implantation procedure is simple. As it is implanted subcutaneously, it reduces the risk of infection. It can be retained for a longer period of time (10 to 20 years). The injection area can be punctured approximately 2000 times, thus avoiding repeated peripheral venous punctures and making it ideal for the intravenous treatment of patients with malignancy [12, 13]. It is easy, safe, and fast to administer medication, simple and convenient to care for, and unrestricted in daily life and bathing. The tube of the implacable IV port needs to be flushed only once in 4 weeks during the nontreatment period. It reduces the number of trips to and from the hospital and the expenses of the patients. Thus, it significantly improves the quality of life of the patients' families. It is a new technology worth promoting, and now, it is the first choice for most oncology patients.

In this paper, we are exploring the role of the smart medical healthcare system architecture and key supporting technologies that are needed to realize this system in a real environment of hospitals. For this purpose, seventy children with hematologic tumors were treated with TIVAP and provided with targeted care, where the occurrence of adverse events, particularly after treatment, was observed. The experimental results after the 70 children were treated and cared for by TIVAP show that there were 5 cases of adverse events, and the incidence rate of adverse events was 7.14%. Thus, TIVAP has significant efficacy in the treatment of pediatric hematologic tumors. Also, it reduces the vascular injury caused by chemotherapy in younger patients, whereas targeted care can reduce the incidence of adverse events in children. The main contributions of this paper are as follows:

- The development of an Internet of Medical Things (IoMT) based smart healthcare system that is designed for the treatment of pediatric hematologic tumors, specifically in children
- To resolve the problem of 100% cure rates per child per day in an effective manner, preferably in the smart healthcare system
- To investigate the clinical application and effectiveness of the completely implantable intravenous port (TIVAP) in pediatric hematologic tumors
- To achieve the expected reduction ratio of pediatric hematologic tumors, particularly in children

The remaining part or sections of our manuscript are organized according to the given format and guidelines. In the subsequent section, the general architecture of the intelligent and smart healthcare system is described in detail.

## 2. Architecture of the Intelligent Medical Healthcare System

The structure of the intelligent medical healthcare system mainly includes the standard specification and security systems that consist of hardware, data, business, exchange four levels, and software. A standard specification system is the data standard that must be followed and managed in the intelligent medical platform. This is the platform operation and application of the database [14, 15]. Security system is used to ensure the normal operation of the whole platform from physical to application. The hardware layer includes hardware devices and network platforms, which constitute the ubiquitous and perception of intelligent medical care. Data layer is mainly to realize the storage of data structure, model, and content. The exchange layer and the business layer mainly realize data collection, exchange, and sharing. The technical layer, which communicates directly with the external systems, is the exchange layer. The business layer is based on the exchange layer and various business service components to achieve the collection, storage, and sharing of platform data.

### 2.1. Implementation Process of the Proposed System

Radio Frequency Identification (RFID) smart shake caller is an extension of the door controller, which is realized by an HF-RFID solution [16]. To ensure 100% reliability of the hospital roll call, a one-to-many approach is used to respond to every individual patient card information assigned to each patient in the smart healthcare system in the form of a card. In other words, an HF reader with multiple antennas is installed in the ward to cycle through all patient cards on the RFID caller.

One of the main contributions of this paper is to solve the problem of 100% cure rates per child per day. The question to be considered now, particularly in this paper, is how to help all the children to enhance their core by high cure rate. The systematic operation or procedure of the proposed mechanism is divided into the following three steps:

  Step 1: the hospital selects this HF card tag as the child's card and preloads all card tag IDs into the hospital's database.
  Step 2: the hospital installs a smart shake in each ward and configures the IP network. The computer central server receives the healing information. In short, each word is realized as an IoT architecture for RFID smart rollers.
  Step 3: remember to bring your child's card. When treating each child, the hospital will look at the child's card to confirm the healing status of each child.

Finally, through these three steps, the hospital will obtain a cure rate for each child. Figures 2 and 3 show a detailed graphical analysis of the proposed mechanism, illustrating how these three steps work interactively, as a general overview of the ward RFID smart roll caller. Figure 1 illustrates the hardware architecture of the RFID smart roll caller.

#### 2.1.1. Hardware Architecture

A new architecture is introduced to collect the correct cure information of each child from each ward in different hospital buildings to confirm their right to learn. The proposed system consists of four main parts: LED display, multi-antenna card slot, card reader module, and embedded system. These parts are described as follows (Figure 3):

  Part 1: LED display that is used by the system to display the child's name and count the number of people in the ward when the child puts the card into the second part.
  Part 2: multiantenna card slots, the system uses these slots to cycle through each RFID patient card and read the tag ID as their patient number to log into the O1 subsystem.
  Part 3: card reader module, the roll call system uses the card reader module to control all antenna card slots and save the patient card ID data to the buffer memory. The card reader module transmits the cure to O1 when O1 leaves the ward.
  Part 4: embedded system is where the system communicates with a computer center server through a LAN environment. In other words, the IP-based roll call system is connected to a switched network.

#### 2.1.2. System Functions

The functions of the roll call system were developed on a server installed in the university computer center using Microsoft VB and .NET programming tools. Microsoft SQL 2018 was used as the database to create and manage the IDs and IPs of the patient cards for the RFID controllers on campus. The three functions and processes of the roll call system are as follows:

- Child Nurse Desk, this subsystem records the cure rate for each child and saves it as the treatment rate for each child. Then, the child and the doctor will receive the last core record from the system at the same time.
- Medical Service, the subsystem calculates the class statistics, departmental statistics, and time period statistics through the system. This real time information will help everyone remember to help the affected child to go to treatment.
- Computer Center, this subsystem manages the installation status of each roll called and sets the configuration of the IP parameters. It also synchronizes the real time clock in each roll-caller and simultaneously sends the healing of each class back to Subsystem-A.

## 3. Internet of Medical Things

The Internet of Medical Things (IoMT) is a collection of various electronics devices, preferably with embedded sensors and actuation modules, to form an operational networking infrastructure, specifically without human intervention.

### 3.1. Sensing Module of the Proposed System

The IoT is mainly used to help the intelligent perception of medical objects (doctors and patients, materials, etc.) to support the digital collection, processing, and storage of equipment, drugs, personnel information, and other information. This information is used to achieve the visualization of medical management, digital information, closed-loop processes, scientific decision-making, and humanized services. Additionally, it is used to solve the problems of weak support, low-level medical safety, etc. In the intelligent medical healthcare systems, the IoT perception system is an important part of the system that enhances the perception of the environment and activities through sensors, RFID, 2D codes, collectors, and other perception technologies and devices to achieve intelligent [17, 18].

### 3.2. Big Data

Big data not only provides scientific basis for single disease diagnosis and treatment but also improves the intelligence of management, decision-making, and evaluation in the medical field. By establishing a big data analysis system based on classification estimation, prediction, association rules, clustering, description, and visualization technologies, we can mine and analyze the huge amount of medical and health big data. The system provides quantifiable decision support for the unified planning and allocation of medical resources, disease occurrence, and epidemic trends, and thus, it improves the management, decision-making, and evaluation in the medical field [19]. At the same time, it also can alleviate the problem of doctor-patient.

### 3.3. Cloud Computing

The application of shared cloud computing expands the commonality of medical resources and services and provides an intelligent, efficient, and highly integrated data sharing platform for intelligent healthcare. Cloud computing distributes services on demand across a pool of resources consisting of a large number of computers. Users can access storage and read data and run software anytime and anywhere using large-scale server clusters on the internet, thus expanding the terminal computing capacity and storage space [20, 21].

### 3.4. Virtual Reality of 3D Holographic Technology

The application of three-dimensional holographic technology has created new changes for surgery, diagnosis, and telemedicine. The application of three-dimensional holographic technology mainly includes two aspects: one is to receive the dimensional holographic data and calculate the hologram; second, the photoelectric system can print or reproduce the image in real space according to the hologram. The real reproduction of 3D holographic technology can replace the previous two-dimensional, clearer observation and analysis of organs and can penetrate, touch, and observe the interaction with the surrounding tissue. It provides great convenience for doctor-patient interaction and surgery [22, 23].

## 4. Proposed Mechanism: Materials and Methods

### 4.1. General Information and Methods

From January 2015 to January 2018, 70 children with hematologic tumors treated with fully implanted intravenous infusion ports in our hospital were selected as observation subjects (inclusion criteria):

1. Children were diagnosed with hematologic tumors according to WHO hematologic tumor diagnostic criteria
2. Children aged 3 to 7 years
3. Children whose parents understood the content of the study and signed the informed consent form

There were 34 male children and 36 female children; age ranged from 3 to 7 years (average 5.36 ± 1.71 years); there were 6 cases of lymphoma, 6 cases of nephroblastoma, 27 cases of neuroblastoma, and 31 cases of leukemia [20].

#### 4.1.1. Implantation Method

Ultrasound-guided internal venous implantation was used, i.e., the catheter was drawn into the ipsilateral clavicle of the child along the subcutaneous path via ultrasound guidance. Moreover, the tip of the catheter was adjusted to the connection of the right atrium and superior vena cave by C-arm fluoroscopy. The infusion port and the catheter were connected, and the infusion port was implanted subcutaneously and closed with sutures. A postoperative X-ray was taken to confirm that the catheter was in the correct position.

#### 4.1.2. Care Methods

Care should be given to children with hematological tumors when implanting infusion ports in the following manner:

1. Preoperative care: preoperative blood routine and coagulation function checks should be performed on the child, and if the child's platelets are lower than 30 × 109/L, platelets should be given before surgery. The parents should be informed of the purpose and significance of TIVAP, postoperative care methods, possible adverse reactions, and preventive measures before surgery to improve their cooperation. The parents should be informed of the purpose of TIVAP, its significance, postoperative care, possible adverse effects, and preventive measures.
2. Intraoperative care: during the operation, adhere to the aseptic procedure and pay attention to the child's posture at all times and make good risk plans. Before pushing the medication to the child, the skin around the injection base should be carefully evaluated for swelling and pus. Then, the injection base should be disinfected three times in a clockwise and counterclockwise manner, and the needle should be punctured with a butterfly-wing needle. At the same time, if the child has no need for infusion for a short period of time, then the tube should be flushed with 20 ml of saline, and subsequently, it has to be sealed with 100 U/L of heparin solutions.
3. Postoperative care and daily care: parents should be instructed to restrict the child from strenuous exercises after the implantation of the intravenous port. The nursing staff should change the child's medication for the first time after 24 hours and pay close attention to the child's vital signs within 3 days.
4. Daily care: the catheter must be thoroughly flushed before and after the infusion, and the bevel of the nondamaging needle should be back to the catheter interface at the base of the infusion port before extraction. The tube must be sealed by positive pressure before extraction to prevent blood reflux. Saline should be flushed at intervals when there is antagonism or incompatibility between the two infusion solutions before and after. The operation related to the infusion port should be strictly aseptic, and once the child shows the symptoms of infection, blood should be taken for poetry dish test first. After the child is discharged from the hospital, an information file on the child's TIVAP should be established (time of implantation, implant type, age of the child, condition, occurrence of adverse reactions, etc.) along with a perfect follow-up system, and a maintenance manual should be issued to the parents with instructions on the maintenance of the TIVAP so that the parents will insist on bringing the child to the hospital every 4 weeks for a heparin-saline flush tube.

### 4.2. Observed Indicators

We have evaluated the effectiveness of TIVAP application and care by observing the incidence of adverse events in the treatment and care of children.

### 4.3. Experimental Results and Observations

After 70 children were treated and cared for with TIVAP, there were 5 adverse events, with an incidence rate of 7.14%, and the distribution of adverse events by age is shown in Table 1.

Furthermore, Figure 4(a) provides the confusion matrix of the root nodes at level 1.  Figure 4(c) shows the clustering of the confusion classes for the healing effect of the affected children obtained by applying the spectrum copolymerization algorithm. We observe three clusters. This clustering can be interpreted as a data hierarchy automatically generated from the affected child data. We fine-tune the network using the IoT architecture, which contributes to the block diagonalization of the confusion matrix. It can be observed from Figure 4 that the use of IoT on the affected children cure effect brings the samples belonging to the same cluster closer, while samples in different clusters were moved further apart. In particular, the use of multivariate analysis improves the robustness of the model classification, and the separation of the affected child cure feature space allows minimizing the connection loss function without affecting the classification performance, which, in fact, shows a slightly improved performance.  Figure 4(b) shows the effect of varying the cluster size *k* on the error rate (due to misclassification); note that the error is minimized when *k* is 3.

The confusion is provided in Figure 5(a). The matrix of root nodes at level 1 and the resulting clusters obtained after applying spectral copolymerization are shown in Figure 5(c). The effect of varying the cluster size *K* on the error rate is shown in Figure 5(b). Even though the error rate is the lowest for *K* = 3, the algorithm selects *K* = 6 for optimal clustering based on the overall fitness. Among these 6 clusters, 3 are composed of a single class in which there is no export network. Needed (since the image classes are already determined). The other three clusters in the image have expert networks of 72, 17, and 8 classes, reducing the classification error for each cluster by more than 10%.

### 4.4. Specific Cases

Mengmeng (pseudonym), 6 years old, presented 20 days ago with no obvious cause for an external supraocular swelling in the right eye, accompanied by multiple skin petechiae. After examination, the diagnosis of acute myeloid leukemia was finally confirmed, and the doctor decided to follow-up with a chemotherapy regimen. Faced with chemotherapy, the family was a bit overwhelmed by the small size of the child, fine blood vessels, and poor cooperation. After being introduced to the doctors and nurses, Mengmeng's mother learned about the relevant vascular accesses, among which, an infusion port could help solve the problem. It is implanted in the child under anesthesia, and all devices are subcutaneously implanted. They can be retained for a long time and maintained once a month. The port does not affect the child's bathing, gets rid of the strange eyes of small partners, does not hurt the child's self-esteem, reduces the child's psychological burden, and significantly improves the quality of life of the child and parents. Mengmeng's parents decided to implant the infusion port for their child. The schematic diagram of body placement in infusion port is as shown in Figure 6.

Our hospital has been using infusion port technology for many years. To standardize this technology and reduce the occurrence of clinical complications, an infusion port MDT team was formed by the hospital's medical office. It is led by the vascular surgery department with the participation of the interventional department and PICC clinic to jointly manage the whole process of infusion port, as shown in Figure 7.

## 5. Discussion

TIVAP is a simple and well-maintained method of drug delivery that protects the patient's blood vessels and significantly improves the quality of life of children with hematomas [1]. Intraoperative care is effective in avoiding venous wall damage and blood hyper coagulation, thus preventing the occurrence of thrombosis. The first drug change 24 hours after the surgery can check the child's body response for infection and other stressful conditions to facilitate the first intervention, whereas close monitoring and informing parents to avoid the strenuous movement of the child can effectively reduce the risk of implant displacement because of the child's body movement. In addition, catheter-associated infections and decreased catheter patency are often caused by the improper maintenance of the port of infusion or failure to follow strict aseptic protocols. Hence, postoperative routine care provides specific requirements for routine maintenance tasks, such as flushing, to ensure that the child is protected from infection and blockage during treatment and that the condition continues to progress well. In addition, according to a survey report [2], approximately 89.42% of the patients' families were not aware of the timing of regular tube flushing after chemotherapy. Hence, the establishment of a TIVAP file and health education for parents after the child's discharge can effectively prevent additional injuries caused by improper parental care or irregular tube flushing. In conclusion, TIVAP can reduce the pain of children and improve their quality of life in the treatment of pediatric hematologic tumors, and it can reduce the incidence of adverse events with targeted care.

## 6. Conclusion and Future Directives

In this paper, we have focused on the role of smart medical healthcare system architecture and key supporting technologies to improve the expected level of traditional treatment carried out in the hospitals. The proposed scheme explores the clinical application and nursing effect of totally implantable intravenous port (TIVAP) in pediatric hematologic tumors and describes how the proposed mechanism is used in speeding up the recovery process of the underlined patients in the hospitals. TIVAP has a significant efficacy in the treatment of pediatric hematologic tumors, and also, it reduces the vascular injury caused by chemotherapy in younger patients. Targeted care can reduce the incidence of adverse reactions in children.

In future, we will explore the potentials of the proposed mechanism in speeding up the recovery process in other diseases as well.

## Figures and Tables

**Figure 1:** The schematic diagram of an infusion port.

**Figure 2:** RFID-roll call architecture.

**Figure 3:** The three functions of the proposed roll-call system's process.

**Figure 4:** Child Results (the best clustering obtained using the Lupin metric is at *K* = 3, which incidentally also corresponds to the lowest misclassification error): (a) the confusion matrix of level 1 nodes, (b) error in the classification of different clusters, and (c) the mirror matrix of different clusters at *k* = 3.

**Figure 5:** Children-doctor Results (even though the misclassification error is the lowest at *K* = 3, the best clusters obtained using the Lupin metric are at *K* = 6. As we expect, i.e., the Lupin metric encourages partitioning into more clusters while keeping the error low): (a) the confusion matrix of level 1 nodes, (b) error in the classification of different clusters, and (c) the mirror matrix of different clusters at *k* = 3.

**Figure 6:** The schematic diagram of body placement in infusion port.

**Figure 7:** The body placement of children in infusion port.

**Table 1:** The occurrence of adverse events in 70 children treated and cared for by TIVAP, *n* (%)).

Adverse reaction	4 years old	5 years old	6 years old	7 years old	Total
Thrombus	0	1	0	0	1 (1.43)
Decreased catheter patency	0	0	0	1	1 (1.43)
Catheter associated infection	0	1	1	0	2 (2.86)
Poor wound healing	1	0	0	0	1 (1.43)

## Data Availability

The datasets used and analyzed during the current study are available from the corresponding author upon reasonable request.
